The article "Fault Diagnosis of Balancing Machine Based on ISSA-ELM" was published in 2022. Journal: Comput Intell Neurosci.

# Fault Diagnosis of Balancing Machine Based on ISSA-ELM

**DOI:** 10.1155/2022/4981022

**Published:** 2022-10-15

**Authors:** Lei Li, Kai Liu, Lei Wang, Li Sun, Zheng Zhang, Hao Guo

**Affiliations:** School of Mechanical Engineering, Jiangsu University of Science and Technology, Zhenjiang 212013, China

## Abstract

Balancing machine is a general equipment for dynamic balance verification of rotating parts, whether it breaks down or does not determine the accuracy of dynamic balance verification. In order to solve the problem of insufficient fault diagnosis accuracy of balancing machine, a fault diagnosis method of balancing machine based on the Improved Sparrow Search Algorithm (ISSA) optimized Extreme Learning Machine (ELM) was proposed. Firstly, iterative chaos mapping and Fuch chaos mapping were introduced to initialize the population and increase the population diversity. Secondly, the adaptive dynamic factor and Levy flight strategy were also introduced to update the individual positions and improve the model convergence speed. Finally, the fault feature vector was input to the ISSA-ELM model with the fault type as the output. The experiment showed that the fault diagnosis accuracy of ISSA-ELM is as high as 99.17%, which is 1.67%, 2.50%, 7.50%, and 17.50% higher than that of SSA-ELM, HHO-ELM, PSO-ELM, and ELM, respectively, further improving the prediction accuracy of the operation state of the balancing machine.

## 1. Introduction

In the machinery manufacturing industry, unbalanced centrifugal forces and centrifugal moments appear in rotating parts (shafts, gears, etc.), which lightly lead to an increase in the load of rotating parts and shorten their service life and seriously cause the generation of fatigue notches in rotating shafts and their mounting parts, causing fractures and endangering personal safety. So, it is essential to correct the dynamic balance of rotating parts. Balancing machine is a common piece of equipment for dynamic balancing calibration of rotating parts, whether its failure occurs or does not determine the accuracy of dynamic balancing calibration. Therefore, it is very meaningful to carry out fault diagnosis for balancing machine.

Extreme learning machine (ELM) is a single hidden layer feedforward neural network [1, 2], which is characterized by simple structure and fast training speed compared with the traditional BP neural network trained based on gradient descent [3, 4]. Therefore, ELM is widely used in the field of fault diagnosis. Lim and Ji [5] apply ELM to fault diagnosis of PV systems. In [6], a new fault diagnosis model for rotating machinery based on residual network (Reset) and ELM is established. In [7], the cuckoo search algorithm (CSA) is introduced to optimize the ELM to achieve the goal of fault diagnosis for fans. In [8], finite element method (FEM) simulation and ELM are combined to detect gear faults. In [9], a multiscale fractal box dimension based on complementary ensemble empirical modal decomposition (CEEMD) and ELM is proposed for planetary gear fault diagnosis.

However, the randomly set weights and biases in ELM affect the computational speed and accuracy of the algorithm, so an optimization algorithm needs to be introduced to optimize the weights and biases to improve the computational efficiency of the algorithm [10]. With the development of machine learning, a large number of swarm intelligence optimization algorithms have been proposed and used. Yang et al. [11] use PSO to optimize the parameters of DBN models and use the optimized DBN models to identify faults. Abbas et al. [12] apply the WOA algorithm to the diagnosis of breast cancer. Han et al. [13] propose a power transformer fault diagnosis model based on HHO optimized KELM. Zhang et al. [14] proposed a fault-detection method based on multiscale permutation entropy and SOA-SVM. The sparrow search algorithm (SSA) [15], as a novel optimization algorithm, is characterized by strong merit-seeking ability and fast convergence compared with traditional swarm intelligence optimization algorithms such as particle swarm algorithm (PSO), and has been applied in a large number of engineering fields. In [16], a new fault diagnosis method based on elite opponent Sparrow search algorithm (EOSEA) optimized LightGBM is proposed. In [17], a deep belief network (DBN) approach based on parameter optimization of SSA is proposed in order to detect gear fault severity. In [18], the signal is decomposed by variational modal decomposition (VMD), and the signal features are extracted by RCMDE and input to the support vector machine (SVM) model optimized by SSA to achieve the fault diagnosis of rolling bearings. In [19], the penalty factor and kernel function parameters of the SVM are optimized using the SSA, and the SSA-SVM wind turbine fault diagnosis model is constructed. In [20], an ELM arc fault diagnosis model optimized by the SSA is developed. However, the SSA algorithm also has the disadvantage of easily falling into local optimum. Therefore, this study proposes an improved SSA algorithm (ISSA) and introduces the ISSA algorithm into the optimization process of weights and thresholds of ELM to construct an ISSA-ELM fault diagnosis model.

The rest of this study is organized as follows.  Section 2 focuses on the principles related to the algorithm.  Section 3 introduces the ISSA-ELM model.  Section 4 describes the experiments. Finally, conclusions are given in Section 5.

## 2. Basic Algorithm Principles

For rotating mechanism such as balancing machine, machine learning is often used to construct fault diagnosis model to analyse its fault. ELM, as a machine learning model, is applied to fault diagnosis by its fast training speed and high accuracy of operation, but the weights and bias in the extreme learning machine are randomly generated, which seriously affect the accuracy of its operation, so the optimization algorithm needs to be introduced to improve the accuracy of ELM, and the standard SSA has the disadvantage of easily falling into local optimum, so the improvement strategy needs to be introduced to improve it.

### 2.1. Sparrow Search Algorithm and Improvement

#### 2.1.1. Sparrow Search Algorithm

The SSA algorithm simulates sparrow foraging and anti-predation behaviors by continuously updating individual positions for the purpose of finding optimal values. In the SSA algorithm, all individuals can be divided into discoverers, followers, and vigilantes.

The update equation for the location of the discoverers is as follows:

(1) $$\begin{array}{c} x_{i,j}^{t+1}=\left\{\begin{array}{c} \begin{array}{cc} x_{i,j}^{t}\cdot \;\exp\;\left(-\frac{i}{\alpha \cdot {iter}_{\max}}\right), & {if\;R}_{2}<ST,\\ x_{i,j}^{t}+Q\cdot L, & if\;R_{2}\geq ST, \end{array}\\ \; \end{array}\right. \end{array}$$

where *t* represents the current iteration number, *x*_*i*,*j*_^*t*^ denotes the position of the ith sparrow in the *j* th dimension in the *t*th generation, *α* ∈ [0,1], *iter*_max_ is the maximum iteration number, *R*_2_ denotes the alarm value, *ST* denotes the safety threshold, *Q* is a random number obeying normal distribution, *L* is a 1 × *di* *m* all-1 matrix, and *di* *m* denotes the dimensionality. When *R*_2_ < *ST*, it means there are no predators around the foraging area and the finders can search for food extensively; when *R*_2_ ≥ *ST*, it means predators appear and all the finders need to fly to the safety area.

The update equation for the location of the followers is as follows:

(2) $$\begin{array}{c} x_{i,j}^{t+1}=\left\{\begin{array}{cc} Q\cdot \;\exp\left(\frac{x_{worst}^{t}-x_{i,j}^{t}}{i^{2}}\right), & \;if\;i>\frac{n}{2},\\ x_{P}^{t+1}+\left|x_{i,j}^{t}-x_{P}^{t+1}\right|\cdot A^{+}\cdot L, & \text{otherwise,} \end{array}\right.\begin{array}{c} ,\\ , \end{array} \end{array}$$

where *x*_*worst*_^*t*^ denotes the position of the individual with the worst fitness value in the *t*th generation, and *x*_*P*_^*t*+1^ denotes the position of the individual with the best fitness value in the *t*+1 generation. A denotes a 1 × *di* *m* matrix with each element in the matrix randomly predefined as -1 and 1, and *A*^+^=*A*^*T*^(*AA*^*T*^)^−1^. When >*n*/2, it means that the *i* follower has low fitness and needs to fly to other regions; when *i* ≤ *n*/2, the follower will forage near the optimal individual *x*_*P*_.

The update equation for the location of the vigilantes is as follows:

(3) $$\begin{array}{c} x_{i,j}^{t+1}=\left\{\begin{array}{cc} x_{best}^{t}+\beta \cdot \left|x_{i,j}^{t}-x_{best}^{t}\right|, & {if\;f}_{i}>f_{g},\\ x_{i,j}^{t}+k\cdot \left(\frac{\left|x_{i,j}^{t}-x_{worst}^{t}\right|}{\left(f_{i}-f_{w}\right)+\varepsilon }\right), & {if\;f}_{i}=f_{g}, \end{array}\right.\begin{array}{c} ,\\ , \end{array} \end{array}$$

where *x*_*best*_^*t*^ denotes the global optimal position in the *t*th generation, *β* is the control step and follows a normal distribution with mean 0 and variance 1, *k* ∈ [−1,1], *ε* is set as a constant to avoid the denominator being 0, *f*_*i*_ denotes the fitness value of the current individual, and *f*_*g*_ and *f*_*w*_ denote the fitness values of the current global optimal and worst individuals. When *f*_*i*_ > *f*_*g*_, it means that the individual is at the periphery of the population and needs to adopt anti-predatory behavior and keep changing its position to obtain higher fitness; when *f*_*i*_=*f*_*g*_, it means that the individual is at the center of the population and it will keep approaching its nearby companions in order to stay away from the danger area.

#### 2.1.2. Improved Population Initialization Method

The distribution of the initial solution in the solution space largely affects the convergence speed and the search accuracy of the algorithm. The SSA algorithm uses random generation to generate the initialized population, and such a way will destroy the diversity of the population. Chaotic sequences have the characteristics of randomness, ergodicity, and regularity [21], which can increase the population diversity and enhance the ability of the algorithm to search globally. In this study, we introduce iterative chaos mapping [22] and Fuch chaos mapping [23] to improve the population initialization. The expressions of iterative chaos mapping and Fuch chaos mapping are shown in formulae (4) and (5):

(4) $$\begin{array}{c} t_{i+1}=\sin\;\left(\frac{b\pi }{t_{i}}\right), \end{array}$$

(5) $$\begin{array}{c} f_{i+1}=\cos\;\left(\frac{1}{f_{i}^{2}}\right), \end{array}$$

where *b* ∈ [0,1].

The steps of the improved population initialization method are as follows:

(1) randomly generate the population *X* = [*x*_1_, *x*_2_, ⋯, *x*_*n*_], where *i* = 1,2, ⋯, *n* and *d* represents the dimensionality.
(2) Let the range of values of the global solution be [*lb*, *ub*], and we generate iterative population *X*_*t*_ and Fuch population *X*_*f*_ according to the following formulae:
  (6) $$\begin{array}{c} X_{t}=lb+\frac{T+1}{2}\cdot \left(ub-lb\right), \end{array}$$
  (7) $$\begin{array}{c} X_{f}=lb+\frac{F+1}{2}\cdot \left(ub-lb\right), \end{array}$$
where *lb* is the upper bound of the search space, *ub* is the lower bound of the search space, and *T* is the chaotic sequence generated by using formulae (4). *F* is the chaotic sequence generated with formulae (5).
(3) combine the populations *X*, *X*_*t*_ and *X*_*f*_ into a new population with the new population *X*_*new*_ = [*X*, *X*_*t*_, *X*_*f*_], find the fitness value of *X*_*new*_, rank the fitness values of the new population individuals in order from smallest to largest, and take the first N optimal initial solutions as the new initial population of sparrows.

#### 2.1.3. Dynamic Adaptive Factor

Like other swarm intelligence algorithms, the SSA algorithm suffers from disadvantages such as poor global search capability and the tendency to fall into local optimality, resulting in insufficient algorithm development. Therefore, the dynamic adaptive weights are therefore improved for the discoverers' position update equations.

The update equation for the location of the discoverers has been improved as follows:

(8) $$\begin{array}{c} x_{i,j}^{t+1}=\left\{\begin{array}{c} \begin{array}{cc} {\lambda \cdot x}_{i,j}^{t}\cdot \;\exp\;\left(-\frac{i}{\alpha \cdot {iter}_{\max}}\right), & R_{2}<ST,\\ \lambda \cdot x_{i,j}^{t}+Q\cdot L, & R_{2}\geq ST, \end{array}\\ \; \end{array}\right. \end{array}$$

where the equation of dynamic adaptive weights *λ* is as follows:

(9) $$\begin{array}{c} \lambda =1-{\left(\frac{t}{i{ter}_{\max}}\right)}^{3}, \end{array}$$

where *t* is the number of current iterations and *iter*_max_ denotes the maximum number of iterations.

The variation curves of dynamic adaptive factors *λ* are shown in Figure 1.

As can be seen from Figure 1, *λ* has larger values at the beginning of the iteration, and the algorithm has stronger global search ability, larger search range and faster convergence, smaller values at the end of the iteration, and stronger local search ability, which can accurately find the global optimal solution.

#### 2.1.4. Levy Flight Strategy

As with other optimization algorithms, standard SSA may fall into local optimal solutions and thus fail to find the global optimal solution. In this study, we introduce the Levy flight strategy [24] to update the position of the vigilantes in the SSA algorithm. The Levy flight strategy is characterized by a long time of small-step random wandering with occasional large steps. The improved SSA algorithm reduces the risk of falling into local optimal solutions. The improved update equation for the location of the vigilantes is shown below:

(10) $$\begin{array}{c} x_{i,j}^{t+1}=\left\{\begin{array}{c} Levy\cdot x_{best}^{t}+\beta \cdot \left|x_{i,j}^{t}-x_{best}^{t}\right|,{if\;f}_{i}>f_{g},\\ x_{i,j}^{t}+k\cdot \left(\frac{\left|x_{i,j}^{t}-x_{worst}^{t}\right|}{\left(f_{i}-f_{w}\right)+\varepsilon }\right),{if\;f}_{i}=f_{g}, \end{array}\right. \end{array}$$

where the equation of Levy flight strategy is as follows:

(11) $$\begin{array}{c} Levy=0.01\cdot \frac{r_{1}\cdot \sigma }{{\left|r_{2}\right|}^{1/\beta }}\text{,}\\ \sigma ={\left\{\frac{\Gamma \left(1+\beta \right)\cdot \;\sin\;\left(\pi \beta /2\right)}{\Gamma \left[\left(1+\beta /2\right)\right]\beta \cdot 2^{\left(\beta -1\right)/2}}\right\}}^{1/\beta }\text{,} \end{array}$$

where Γ is a gamma function, *β* is a constant, taken as 1.5, and *r*_1_ and *r*_2_ are random numbers from 0 to 1.

### 2.2. Extreme Learning Machine

ELM is a fast learning algorithm, which obtains the corresponding output weights by randomly initializing the input weights and offsets [25, 26]. The ELM network structure is shown in Figure 2. The mathematical expression of elm can be expressed as follow:

(12) $$\begin{array}{c} \beta \cdot g\left(W\cdot X+b\right)=T, \end{array}$$

where *g*(*x*) is the activation function, *W* is the input weight, *β* is the output weight, *b* is the hidden layer offset, *X* is the input vector, and *T* is the output vector. Let *g*(*W* · *X*+*b*)=*H*. Then, formulae (13) can be obtained:

(13) $$\begin{array}{c} H\beta =T, \end{array}$$

where *H* is the output matrix of the hidden layer, *β* is the output weight, and *T* is the desired output. The learning process of ELM has the following main steps.

1. We determine the number of neurons in the hidden layer and randomly set the connection weights *ω* between the input layer and the hidden layer and the bias *b* of the neurons in the hidden layer
2. We select an infinitely differentiable function as the activation function of the hidden layer neurons and then calculate the hidden layer output matrix H
3. We calculate the output layer weights *β*=H^+^T, where H^+^ is the Moore–Penrose generalized inverse matrix of H

## 3. ISSA-ELM Modeling

The weights *ω* and bias *b* of ELM are set randomly [27], which seriously affects the accuracy and speed of the algorithm's operation. In this study, an ISSA algorithm is introduced into the process of selecting the ELM weights *ω* and bias *b*, and an ISSA-ELM model is proposed. The method uses the ISSA algorithm to optimize the weights *ω* and bias *b* of ELM, and the weights *ω* and bias *b* in ELM are used as the population individuals in the ISSA algorithm, and the classification error rate of ELM is used as the fitness function to globally search for the optimal value. The ISSA-ELM fault diagnosis flowchart is shown in Figure 3, and the modeling steps are as follows:

1. We set ELM-related parameters.
2. We set the ISSA-related parameters as well as the fitness function. The relevant parameters of ISSA to be set include the maximum number of iterations, the ratio of discoverers, followers and vigilantes, and the population size according to the weights and deviations of ELM. The classification error rate is chosen as the fitness function.
3. We initialize the population. A modified population initialization method is used to generate populations.
4. We calculate initial fitness values and rank them and the fitness value of each individual in the population and rank the individuals in order from smallest to largest fitness value.
5. Sparrow individual position update: we update the discoverers, followers, and vigilantes' positions according to formulae (8), (2), and (10).
6. We calculate the fitness value of the individual after updating the position and determine whether the termination condition is satisfied or the maximum number of iterations is reached; if it is satisfied, the optimal weight and bias are output, if not, we iterate through the loop until the termination condition is met or the maximum number of iterations is reached.
7. The ISSA-ELM model is constructed using the obtained optimal weights and biases.
8. We evaluate the performance of the ISSA-ELM model.

## 4. Experiments

### 4.1. Sample Selection and Feature Extraction

In this study, the fault diagnosis experiment is carried out by using Dewesoft data acquisition system and HY40WUB type hard support balancing machine. As shown in Figure 4, the experiment installs single-phase vibration sensors in the *X*-axis and *Y*-axis directions of the support frame of HY40WUB hard support balancing machine and collects vibration signals through Dewesoft acquisition instrument with a frequency of 2560 HZ. We separate acquisition of fault signals under eight operating conditions of balancing machines.

We extract the fault feature quantity that can reflect the working state of the balancing machine from the *x*-axis and *y*-axis, as shown in Table 1. To remove the influence of different magnitudes, the fault data are normalized according to formulae (14). The feature vectors are obtained, and each group of feature vectors is 44-dimensional. Each class of sample data is 50 groups, totaling 400 sets of fault data, of which 280 groups are used as the training set and 120 groups are used as the test set. The fault types of balancing machine are numbered as 1–8, which are divided into 8 types: normal, belt deterioration, universal coupling wearing, universal coupling rusting, journal abrasion, roller outer diameter wearing, roller outer diameter breakage, and roller rusting. The distribution of sample capacity of training set and test set is shown in Table 2:

(14) $$\begin{array}{c} x^{*}=\frac{x-x_{\min}}{x_{\max}-x_{\min}}, \end{array}$$

where *x*^*∗*^ is the normalized data, *x* is the original data, *x*_max_ is the maximum value in the original data set, and *x*_min_ is the minimum value in the original dataset.

From Table 1, *N* is the number of sampling points, *x*_*i*_ is the *i*th element of any sample in the vibration data set, *f*_*i*_ is the frequency instantaneous value at moment *i*, and *F*(*f*_*i*_) is the Fourier spectrum instantaneous value at moment *i*.

### 4.2. Define the ELM Network Structure

According to the dimension of the input and output quantities, the number of nodes at the input of ELM can be determined as 44 and the number of nodes at the output as 1. The selection of the number of nodes in the hidden layer affects the accuracy of ELM classification, and this study calculates the train accuracy of ELM for the cases of the number of nodes in the hidden layer from 1 to 200, respectively, and the graph of the number of nodes in the hidden layer and the train accuracy is shown in Figure 5.

From Figure 5, it can be seen that the train accuracy of the activation function “sigmod” is higher than that of “sin” and “hardlim”. Therefore, the “sigmod” type function is chosen as the activation function in this study. When the number of nodes in the implied layer is 90∼140, the train accuracy is higher than other ranges. The number of nodes in the implied layer is set to 90, 100, 110, 120, 130, and 140, respectively, and 10 tests are conducted, and the results are shown in Figure 6.

It can be seen from Figure 6 that when the number of ELM nodes is 100, the accuracy rates are all higher than the other node numbers. Therefore, the number of nodes in this study is set to 100.

### 4.3. Analysis of Experimental Results

#### 4.3.1. Performance Comparison of Optimization Algorithms

The adaptation curves of ISSA, SSA, HHO, and PSO to the ELM optimization parameters are shown in Figure 7. The parameters of the four algorithms are set as follows: the maximum number of iterations of ISSA is set to 50, the population size is 20, the proportion of discoverers is 0.2, the proportion of joiners is 0.8, the proportion of vigilantes is 0.1, and the early warning value is set to 0.6; the maximum number of iterations of SSA is set to 50, the population size is 20, the proportion of discoverers is 0.2, the proportion of joiners is 0.8, the proportion of vigilantes is 0.1, and the early warning value is set to 0.6; the maximum number of iterations of HHO is set to 50, the population size is 20; the maximum number of iterations of PSO is set to 50, the particle population size is 20, the inertia factor is set to 0.9, and the acceleration constants c1 and c2 are both 2.

From the fitness curves in Figure 7, it can be seen that the fitness values of all four algorithms start to decrease and converge as the number of iterations increases, so as to obtain the best weights and biases. The initial fitness values are sorted from lowest to highest as ISSA, SSA, HHO, PSO, and ISSA has the lowest initial fitness value; ISSA converges at about the 8th generation, SSA converges at about the 21st generation, HHO converges at about the 26th generation, and PSO converges at about the 29th generation; ISSA finds the optimal solution in the shortest time and converges the fastest; the final convergence fitness values of the four algorithms are ISSA, SSA, HHO, and PSO in the order from smallest to largest, and ISSA has the smallest final fitness value. Therefore, ISSA has the most obvious optimization for ELM.

#### 4.3.2. Comparison of Fault Diagnosis Models

The fault characteristic quantities are input to the ISSA-ELM, SSA-ELM, HHO-ELM, PSO-ELM, and ELM diagnostic models, and the diagnostic time and accuracy are shown in Table 3; the diagnostic results are shown in Figure 8.

In Figure 8, the blue circles represent the actual fault types, the red diamonds represent the fault categories predicted by different models, the horizontal coordinates are the diagnostic sample numbers, and the vertical coordinates are the fault category labels. From Table 3 and Figure 8, it can be seen that ISSA-ELM correctly predicts 119 balancing machine faults with 99.17% fault diagnosis accuracy, which has the highest fault diagnosis accuracy compared with the other four diagnostic models. The results show that the comprehensive fault diagnosis model established by the ISSA algorithm by seeking the weights and biases of ELM can effectively improve the fault diagnosis accuracy of balancing machine.

## 5. Conclusion

To address the problem that the fault diagnosis accuracy of balancing machine needs to be improved, this study proposes a fault diagnosis method based on ISSA-ELM and compares it with SSA-ELM, HHO-ELM, PSO-ELM, and ELM, and the following conclusions can be drawn:

1. The introduction of the iterative chaos mapping and the Fuch chaos mapping to improve the population initialization method can increase the population diversity and enhance the algorithm's global optimization seeking ability
2. The use of dynamic adaptive factor and Levy flight strategy to improve the position update formula of SSA algorithm can effectively improve the disadvantage that SSA algorithm is easy to fall into local optimum
3. Using ISSA algorithm to find the optimal values of weights and thresholds of ELM, the results show that the diagnostic accuracy of ISSA-ELM is higher compared with SSA-ELM, HHO-ELM, PSO-ELM, and ELM, reaching 99.17%, which obviously improves the diagnostic efficiency

In fault diagnosis, multisource information fusion can take into account multiple signals, which can further improve the accuracy of fault diagnosis; therefore, multisource information fusion of balancing machines will be further investigated in future work.

## Figures and Tables

**Figure 1:** Dynamic adaptive factor *λ* variation curve.

**Figure 2:** ELM network structure.

**Figure 3:** Flowchart of the ISSA-ELM fault diagnosis model.

**Figure 4:** Signal acquisition diagram.

**Figure 5:** Comparison of common excitation functions of ELM.

**Figure 6:** Comparison of the number of nodes in the ELM implicit layer.

**Figure 7:** Adaptation curve.

**Figure 8:** Results of fault diagnosis. (a) Results based on ISSA-ELM. (b) Results based on SSA-ELM. (c) Results based on HHO-ELM. (d) Results based on PSO-ELM. (e) Results based on ELM.

**Table 1:** Fault features.

Description	Features
Maximum	*x*_max_=max (*x*_*i*_)
Minimum	*x*_min_=min(*x*_*i*_)
Mean	$\bar{x}=\frac{1}{N}\sum_{i=1}^{N}x_{i}$
Absolute mean	$x^{\prime }=\frac{1}{N}\sum_{i=1}^{N}\left|x_{i}\right|$
Square root amplitude	$x_{s}={\left(1/N\sum_{i=1}^{N}\sqrt{\left|x_{i}\right|}\right)}^{2}$
Peak-peak value	*x*_*p*−*p*_=max(*x*_*i*_) − min (*x*_*i*_)
Variance	$\delta =1/N\sum_{i=1}^{N}{\left(x_{i}-\bar{x}\right)}^{2}$
Standard deviation	$\sigma_{x}=\sqrt{1/N-1\sum_{i=1}^{N}{\left(x_{i}-\bar{x}\right)}^{2}}$
Kurtosis	*β*=1/*N*∑_*i*=1_^*N*^*x*_*i*_^4^
Skewness	*α*=1/*N*∑_*i*=1_^*N*^*x*_*i*_^3^
Mean square	*x*_*ms*_=1/*N*∑_*i*=1_^*N*^*x*_*i*_^2^
Root mean square	$x_{rms}=\sqrt{1/N\sum_{i=1}^{N}x_{i}^{2}}$
Waveform factor	*W*=*x*_*rms*_/*x*′
Peak factor	*C*=*x*_max_/*x*_*rms*_
Pulse factor	*I*=*x*_max_/*x*′
Margin factor	$L=x_{rms}/\bar{x}$
Kurtosis factor	*K*=*β*/*x*_*rms*_^4^
Frequency of center of gravity	*x*_*fc*_=∑_*i*=1_^*N*^*f*_*i*_*F*(*f*_*i*_)/∑_*i*=1_^*N*^*F*(*f*_*i*_)
Mean square frequency	*X*_*msf*_=∑_*i*=1_^*N*^*f*_*i*_^2^*F*(*f*_*i*_)/∑_*i*=1_^*N*^*F*(*f*_*i*_)
Root mean square frequency	$X_{rmsf}=\sqrt{\sum_{i=1}^{N}f_{i}^{2}F\left(f_{i}\right)/\sum_{i=1}^{N}F\left(f_{i}\right)}$
Frequency variance	*X*_*vf*_=∑_*i*=1_^*N*^(*f*_*i*_ − *X*_*fc*_)^2^*F*(*f*_*i*_)/∑_*i*=1_^*N*^*F*(*f*_*i*_)
Frequency standard deviation	$X_{rvf}=\sqrt{\sum_{i=1}^{N}{\left(f_{i}-X_{fc}\right)}^{2}F\left(f_{i}\right)/\sum_{i=1}^{N}F\left(f_{i}\right)}$

**Table 2:** Sample size distribution.

Fault number	Fault type	Training samples	Test samples
1	Normal	35	15
2	Belt deterioration	35	15
3	Universal coupling wearing	35	15
4	Universal coupling rusting	35	15
5	Journal abrasion	35	15
6	Roller outer diameter wearing	35	15
7	Roller outer diameter breakage	35	15
8	Roller rusting	35	15

**Table 3:** Calculation results of different algorithms.

Fault number	Fault type	Fault recognition number				
		ISSA-ELM	SSA-ELM	HHO-ELM	PSO-ELM	ELM
1	Normal	15	15	14	15	14
2	Belt deterioration	14	12	12	11	8
3	Universal coupling wearing	15	15	15	15	13
4	Universal coupling rusting	15	15	15	15	10
5	Journal abrasion	15	15	15	13	13
6	Roller outer diameter wearing	15	15	15	13	13
7	Roller outer diameter breakage	15	15	15	13	12
8	Roller rusting	15	15	15	15	15
Accuracy		99.17%	97.50%	96.67%	91.67%	81.67%

## Data Availability

The data used to support the findings of this study can be obtained from the corresponding author upon request.
